# Study on Allopathic and Alternative Treatments of Asthma and Factors Influencing Treatment Choices

**DOI:** 10.1155/2022/4699414

**Published:** 2022-08-29

**Authors:** Javeria Farooq, Sheikh Abdul Khaliq, Faiza Ghuman, Javeria Shaikh, Iqbal Azhar

**Affiliations:** ^1^Faculty of Health Sciences, Iqra University, Karachi, Pakistan; ^2^Department of Pharmacy Practice and Pharmaceutics, Faculty of Pharmacy, Hamdard University, Karachi 74600, Pakistan; ^3^Department of Medicine, Dow University of Health Sciences, Karachi, Pakistan; ^4^Department of Pulmonology, Dow University of Health Sciences, Karachi, Pakistan; ^5^Faculty of Pharmacy and Pharmaceutical Sciences, University of Karachi, Karachi, Pakistan

## Abstract

**Materials and Methods:**

The cross-sectional survey was conducted; primary data were collected from asthmatic patients in different hospitals and clinics of allopathic, homeopathic, and herbal practitioners in Karachi, Pakistan. The study duration was from January 2020 to December 2020. Asthmatic patients aged over 13 years were selected for the study. A written informed consent was taken from the patients before the interview. Collected data were analyzed by the Statistical Package of Social Sciences (SPSS) 22.

**Result:**

Among 255 asthmatic patients; 51.4% (*n* = 131) were male and 48.6% (*n* = 124) were female. For control of acute attacks of asthma 88.2% (*p* = 0.0001) of patients significantly preferred allopathic treatment while 6.3% (*p* = 0.008) used homeopathic treatment and 5.5% chose herbal treatment. For maintenance of asthma, 78.8% (*p* = 0.0001) patients used allopathic treatment while 12.4% (*p* = 0.0001) homeopathic and 8.8% (*p* = 0.0001) patients used herbal treatment. About 63.4% (*p* = 0.0001) of the asthmatic patients used short-acting *β*-2 agonists for managing acute asthmatic episodes while long-acting *β*-2 agonists (*p* = 0.0001) and inhaled corticosteroids (*p* = 0.0001) were found to be the preferred medicines for maintenance therapy. Effectiveness of treatment (*p* = 0.004) and cost effectiveness (*p* = 0.0001) significantly act as contributing factors for the selection of the treatment. The majority of the patients were satisfied with their chosen treatments for control of asthmatic symptoms.

**Conclusion:**

Most asthmatic patients preferred allopathic treatment for the management of acute episodes and control of asthmatic symptoms. It was found that the major factors for selecting a specific treatment include effectiveness, cost, and minimal side effects.

## 1. Introduction

Asthma is a chronic inflammatory disorder [1]. It causes a high global burden of death and disability; around 1000 people die from asthma each day. [1] The prevalence of asthma across Asia ranges from 0.7% to 11.9% [2]. In Pakistan, over 10% of the population is a victim of asthma [1]. The largest city in Pakistan is Karachi; about 8–10% population of this mega city suffers from chronic asthma [3]. In addition, asthma is also associated with a significant socioeconomic burden [4]. Such a burden is due to costs of asthma medications, physician's visits, hospital admissions, absence from work, and premature death. Asthma interferes significantly with daily life [5] and limits a patient's physical activities due to asthmatic symptoms. Increased levels of anxiety, fear, and depression also enhance the emotional burden [6]. On the other hand, if asthma is effectively controlled, quality of life might improve and reduce the socioeconomic burden [7]. Proper control of severe asthma prevents exacerbations and limits mortality [1]. Asthma exacerbations might also result due to exposure to a number of risk factors/triggers including allergens, pollutants, smoking, pets, coexisting medical conditions, and medications. Identification and prevention of asthma triggers reduce exacerbation and help in achieving better control [8]. Traffic-related air pollution, nitrogen dioxide, and second-hand smoking exposures represent significant risk factors for asthma development in children [9]. Climate change and air pollution have a significant impact on human health and the onset and aggravation of allergic rhinitis and asthma in patients with chronic respiratory diseases [10]. More than 90% population lives in places where air quality does not meet the recommendation of the World Health Organization; due to this reason, prevalence of asthma is rising in urban areas [11].

Several types of treatments are used to maintain asthma including allopathic and alternative treatments. The allopathic method includes a wide range of drugs such as corticosteroids, short- or long-acting *β*-2 agonists, anticholinergics, bronchodilators, immunomodulators, leukotriene modifiers, mast cell stabilizers, and xanthine-oxidase inhibitors [12]. Immunotherapy or allergy shots improve asthma control in some patients; a recent meta-analysis demonstrated that immunotherapy may improve lung function, reduce symptoms, and decrease medication requirements in a significant number of patients [13]. Diverse treatment approaches with reliever medications, controllers, and combination medications are used for asthma. Unlike other medications, biologicals are also used for the management of asthma in a physician's office. Currently, there are five approved biological for the management of asthma such as omalizumab, mepolizumab, reslizumab, benralizumab, and dupilumab [14]. Omalizumab is an anti-IgE monoclonal antibody compound; it is used for severe asthma and concurrent allergies. It is usually administered twice monthly as an injection in a specialty physician's office. Life-threatening anaphylaxis has rarely been reported with this medication [15]. Systematic reviews of all these five biological agents found that they reduce asthma exacerbation rates with high certainty [14]. The addition of these biological agents is a marked therapeutic advancement, especially for refractory asthma. These agents are licensed for eosinophilic asthma. These biological agents target the Th-2 pathway of cytokines, such as mepolizumab and reslizumab (IL-5), benralizumab (IL-4), and dupilumab (IL-3) [16]. The use of specific approach depends upon the need (acute or maintenance), asthma severity, and patient requirements [17]. In addition to allopathic treatments, many patients use complementary and alternative medicines (CAMs). CAMs are a group of various medical and healthcare approaches, practices, and products not commonly considered a part of conventional medicine. The documented prevalence rates of CAM practice in treating asthma is from 4% to 79% [18]. The common CAM used for asthma includes herbal and homeopathic medications. Herbal medicines are part of the traditional medical practice that uses several plant resources for prevention and therapeutic purpose. Herbal medicines are generally considered as a safe treatment for different diseases and are assumed to be relatively less toxic [19]. Other than commercially available herbal medicines, plants and herbs are also used for asthma including honey, garlic, turmeric, bitter gourd, linseed, and mustard oil [20]. Homeopathy is one of the most common and debated methods of complementary medicine used to treat asthma. Homeopathy identifies disease as a holistic issue and tries to treat the disease from the core rather than focusing on symptoms only [21].

Considering such diversity in the treatments, the primary end-point of the current study was to determine the prevalence of allopathic, homeopathic, and herbal treatments for addressing both acute onsets of asthma and its maintenance. The secondary end-point of the study was to explore which treatment is preferred by patients and which specific class of drug is mostly used for acute asthmatic attacks and for maintenance of relief from asthma.

## 2. Materials and Methods

The survey design was cross-sectional and observational. The multicenter study was conducted at government hospitals, private hospitals, and clinics in the mega city of Pakistan, Karachi. The duration of the study was from January 2020 to December 2020. The sample size of the study was calculated by the precision analysis technique [22]. All study work was conducted in accordance with the Declaration of Helsinki. Ethical approval of the study has been obtained from the Institutional Bioethics Committee, University of Karachi, with approval No. IBC-KU-24. The study was also approved by the Advanced Studies and Research Board, University of Karachi, with approval No. ASRB/02032/Pharm.

After ethical approval, a structured questionnaire was used for the primary data collection. The questionnaire was finalized after multiple iterations and pilot testing in the field. The questionnaire was both in English and Urdu language for a better understanding. Asthmatic patients of age above 13 years were selected for the study. Written informed consent was taken from every participant before the interview, and the questionnaire was completed through face-to-face interviews.

The primary end-point of the current study was to determine the prevalence of allopathic, homeopathic, and herbal treatments for addressing both acute onsets of asthma and its maintenance. The secondary end-point of the study was to explore which treatment is preferred by patients and which specific class of drug is mostly used for acute asthmatic attacks and for maintenance of relief from asthma. By considering these end-points of study, information obtained from the questionnaire included demography of patients such as patient's age, gender, type of asthma, asthma severity, and choice of treatment with conventional/alternative medicines for both acute episodes of asthma and maintenance of relief from asthma. They were also requested to highlight factors that determined their choice of a particular treatment and their satisfaction level with the treatment.  Figure 1 represents the flowchart of the study.

Data confidentiality was maintained and coded to maintain the privacy of participants and consent. Collected data for the study were analyzed by the SPSS (Statistical Package of Social Sciences) version 22. The responses for different groups were compared using the Chi-square test and Friedman test. Any result with a *p* < 0.05 was considered as significant for this study.

## 3. Result

In the survey, a total of 255 asthmatic patients were interviewed.  Table 1 mentioned the frequency and percentage of different characteristics of respondents while a clinical picture of respondents is mentioned in Table 2.

Respondent's treatment preferences and satisfaction levels are shown in Table 3. Respondent's drug preferences for acute asthmatic attacks and maintenance of relief are mentioned in Figures 2 and 3.

Short-acting *β*-2 agonist (SABA) was found to be the most prescribed and statistically significant (*p*=0.0001) drug for the treatment of acute asthmatic episodes and was used by 63.4% of the patients.

For maintenance of relief from asthma, long-acting *β*-2 agonist (LABA) was used by 40.1% of the patient (*p*=0.0001), while 28.4% used ICS/OCS (inhaled/oral corticosteroids) (*p*=0.0001) and 11.0% used leukotriene modifiers (*p*=0.011). In addition, herbal medication/remedies (*p*=0.0001) were used by 12.9% and homeopathic medications (*p*=0.0001) were used by 4.3% of the asthmatic patients.

The survey respondents were also asked about the factors that determine the choice of their respective treatments for acute asthmatic episodes and maintenance of relief from asthma. The different factors included effectiveness of treatment, cost effectiveness, minimal side effects, and easy long-term management among others. Effectiveness of treatment (*p*=0.004) and cost of treatment (*p*=0.0001) were found to be the most significant factors for patients in making treatment choices as shown in Figure 4.

## 4. Discussion

The findings of the study were consistent with the hypothesis of the study; the majority of the patients interviewed at different centers all over Karachi preferred allopathic treatment for controlling the acute attack of asthma. Very few patients choose homeopathic and herbal treatments for acute asthmatic attacks. Similarly, for controlling the chronic symptoms of asthma, the patients also preferred allopathic treatment compared to homeopathic and herbal treatments. The current study validated that allopathic is a more effective and trustworthy treatment for asthma as compared to homeopathic and herbal treatments. Some literature presented that homeopathy plays a major role in the management of asthma both in acute and chronic asymptomatic phases [23]. It reduces the use of allopathic/conventional drugs [23]. However, randomized trials are mandatory to validate the efficacy of homeopathy in asthma. In addition to randomized trials, observational studies are also necessary to determine the homeopathic drugs prescribed and the patient's response [23]. Herbal treatment has been found to be an effective alternative treatment for asthma, but still, for the safe and effective prescription of herbal medications evidence-based studies, particularly clinical trials are required [24].

The current study reveals that patients preferred homeopathic and herbal treatments for controlling chronic symptoms of asthma as compared to acute attacks. Such findings increased reliance on homeopathic and herbal treatments for controlling chronic symptoms, which is in line with the findings of Clarke et al., where they found that because of the risk of possible adverse effects pertaining to long-term use of allopathic medications; many patients avoid allopathic or conventional medicines. Furthermore, nonadherence to conventional (allopathic) treatment might be due to complex treatment regimens and difficult inhalation techniques [19]. A study also found that improper use of inhalers affects the quality of life of an asthmatic patient and also results in nonadherence to allopathic treatment [25].

The current study data showed that from available and prescribed medications including allopathic, herbal, and homeopathic, the short-acting *β*-2 agonist is used by most of the patients for acute asthmatic episodes while the second most used drug was inhaled corticosteroid. For maintenance of relief from asthma, long-acting *β*-2 agonist and inhaled/oral corticosteroid were the preferred choices by asthmatic patients. The study findings are in line with previous findings; most asthmatic patients used short-acting *β*-2 agonist as a first-line treatment for acute asthmatic attacks [26] and provides quick relief from symptoms [27]. Controlling chronic symptoms of asthma, responses of the patients also coincided with the recommended guidelines that long-acting *β*-2 agonists and inhaled corticosteroids [28] are an effective treatment for long-term relief from asthma. It was also noted that some of the respondents were using both long-acting *β*-2 agonists and inhaled corticosteroids for relief from asthmatic symptoms; such a combination is reported to be effective in asthma control and preventing exacerbations [29]. These treatment preferences also strengthen the patient's response that the main factor for selecting a specific treatment or medication is the effectiveness of the treatment. Route of drug administration might be another major contributing factor to the preference of patients for allopathic medicines. The survey findings verified that most of the medications used for asthma control belong to the allopathic medicine system; the inhalation route is found to be the most effective one with rapid onset of action for respiratory disorders [30].

The results of this study also showed that most of the patients using different treatments were satisfied with their chosen treatment for both acute attacks of asthma as well as for chronic relief from asthma. Although homeopathic and herbal treatments were used by a small number of patients, most of them were satisfied with their treatment for both acute and chronic relief. It shows that allopathic was the preferred treatment for asthma; however, homeopathic and herbal treatments were also found to be effective for both reducing acute asthmatic episodes and for chronic relief. These findings are contradictory to the results of Chen et al., which showed that the use of alternative and complementary therapies is associated with a lack of asthma control. However, the study also included many alternative treatments other than homeopathic and herbal treatments [18].

The study also focused on factors that patients considered important when choosing treatment for asthma. The majority of respondents rank the effectiveness of treatment as the most important factor for the choice of treatment type. In addition, the cost of treatment is also significantly considered by respondents while selecting a treatment. It was observed that patients understand the fact that asthma is a chronic disease, so they also consider minimal side effects and easy long-term management before choosing a treatment. These findings of the study validate that allopathic is the most preferred treatment for asthma in terms of efficacy. The efficacy of allopathic medication has been proven by many research studies. However, current study results also support the outcome of Herman and his colleagues' study that further analysis of cost effectiveness should be performed on alternative treatments [31].

Another important finding of this study suggests that patients' basic needs are the positive outcome with any of the treatments they select. Patient preference or choice of a specific treatment may also be affected by many psychological factors such as motivation to recover; attitude towards asthma; the medication; the prescriber; attitudes; and views of surrounding individuals [32]. Various studies evaluated the role of the health care provider which holds a very significant position and can affect the patient's decision of acceptability to the treatment. If the exacerbated presentation of specific treatment benefits including efficacy, better tolerance, cost, and fewer side effects is presented by health care providers, it will definitely increase the adherence of patients to the prescribed treatment [33, 34]. It is also necessary to highlight the increasing prevalence of alternative treatments; physicians, pharmacists, and clinicians should have knowledge and information to guide their patients about the use, benefits, and possible side effects of alternative therapies [35]. Physicians should regularly evaluate the triggers for individual patients, and support and educate patients to manage the effect of asthma triggers [36]. Pharmacists can also play a significant role in the education of patients about the disease as well as the types of drugs used.

## 5. Conclusion

The study found that allopathic treatment is the most preferred treatment for both acute asthmatic attacks and relief from chronic asthma. Effectiveness and cost of the treatment were the key factors for selecting a particular treatment. The findings of the study may provide a way forward for understanding patients' values and preferences regarding their treatment and enhancing their satisfaction levels.

## 6. Recommendations

It is important that any treatment provided by healthcare providers should be prescribed only after the identification of a moderate, severe, or life-threatening exacerbation. They should always first identify the symptoms, signs, and risk factors for severe and life-threatening exacerbations and then prescribe treatment that is better for patients in terms of effectiveness, safety, and economy. The ECHO (economic outcome, clinical outcome, and humanistic outcome) model should be applied. [37] Evidence-based studies and randomized clinical trials are required to confirm the efficacy and safety of alternative treatment methods for asthma in order to use them more with allopathic medications.

## Figures and Tables

**Figure 1:** Study flowchart.

**Figure 2:** Drug preference for acute asthma episode. SABA: short-acting *β* agonist; ICS: inhaled corticosteroids; LABA: long-acting *β* agonist. Results are presented as a percentage with *p* value < 0.05.

**Figure 3:** Drug preference for asthma maintenance. ICS: inhaled corticosteroids; OCS: oral corticosteroids; LABA: long-acting *β*-2 agonist. Results are presented as a percentage with *p* value < 0.05.

**Figure 4:** Factors affecting the choice of treatment in asthma. Results are presented as a percentage with *p* value < 0.05.

**Table 1:** Characteristics of respondents.

Variables	Groups	Frequency	
		*N*	%
Gender	Male	131	51.57
	Female	123	48.43

Age	14–24 years	34	13.44
	25–34 years	40	15.81
	35–44 years	58	22.92
	45–54 years	51	20.16
	55–64 years	40	15.81
	65 years or older	30	11.86

Education	No formal education	57	22.53
	Primary	38	15.02
	Secondary	36	14.23
	Intermediate	35	13.83
	Graduate	56	22.13
	Masters/Professionals	31	12.25

Work	Yes	116	45.85
	No	137	54.15

Income	Up to rs 10,000	55	22.54
	Rs 10,000–25,000	84	34.43
	Rs 25,000–50,000	44	18.03
	Rs 50,001–75,000	19	7.79
	Rs 75,001–100,000	18	7.38
	Above rs 100,000	24	9.84

Smoking	Yes	55	21.83
	No	197	78.17

Smoker in family	Yes	85	34.14
	No	164	65.86

Pets	Yes	114	44.88
	No	140	55.12

Surroundings	Clean residence	120	47.06
	Garbage near residence	101	39.61
	Water standing around the residence	59	23.14
	Construction near residence	43	16.86
	Highly populated residence	48	18.9

**Table 2:** Clinical picture of respondents.

Variables	Groups	Frequency	
		*N*	%
Age while asthma was diagnosed	Under the age of 14 years	57	24.8
	15–24 years	62	27.0
	25–34 years	53	23.0
	35–44 years	37	16.1
	45–54 years	9	3.9
	55–64 years	9	3.9
	65 years or older	3	1.3

Symptoms	Cough	179	70.2
	Wheezing	123	48.2
	Chest tightness	165	64.7
	Shortness of breath	195	76.5
	Phlegm production	91	35.7

Severity	Intermittent	106	41.6
	Mild	88	34.5
	Moderate	50	19.6
	Severe	11	4.3

Limitation in daily life due to asthma	Minor/No limitation	138	55
	Some limitation	86	34.3
	Extremely limited	27	10.7

**Table 3:** Treatment preferences and satisfaction level of respondents.

Variables	Groups	Allopathic		Homeopathic		Herbal	
		%	*p* value	%	*p* value	%	*p* value
Asthma	Acute	88.2	0.0001	6.3	0.008	5.5	0.057
	Maintenance	78.8	0.0001	12.4	0.001	8.8	0.0001
	Not satisfied at all	—		—		—	

Satisfaction level (acute)	Not satisfied	6		—		8	0.015
	Neutral	20	0.008	20	0.284	8	
	Satisfied	62		80		76	
	Extremely satisfied	12		—		8	

Satisfaction level (maintenance)	Not satisfied at all	—		—		5	0.0001
	Not satisfied	6		8		5	
	Neutral	19	0.373	11	0.232	14	
	Satisfied	63		70		71	
	Extremely satisfied	12		11		5	

## Data Availability

The datasets generated during the current study are not publicly available to maintain the confidentiality of participants but are available from the corresponding author on a reasonable request.
